# HPLC Analytical Method Development and Validation of Gabapentin through Chemical Derivatization with Catechol as a Chromophore

**DOI:** 10.1155/2022/3882682

**Published:** 2022-10-03

**Authors:** Murad Abualhasan, Fairouz Shraim, Hiba Alawni, Saba Hamdan, Hadeel Khaseeb

**Affiliations:** Department of Pharmacy, Faculty of Medicine & Health Sciences, An-Najah National University, Nablus, State of Palestine

## Abstract

**Background:**

Gabapentin is a drug with anticonvulsant activity and has been widely used in the treatment of epilepsy. Gabapentin chemical structure lacks a chromophore which makes its absorption very low and hence complicates its analysis and reduces the sensitivity of the method. Adding a chromophore by chemical derivatization makes the drug easily identified and quantified at a much lower concentration using chromatographic analysis such as HPLC. *Methodology*. The derivatization of gabapentin was done by adding a chromophore to the structure by introducing an auxochrome group. Suitable coupling reagents were used to introduce catechol group to gabapentin. The analytical method has been developed using HPLC with UV/Vis detector. Moreover, the method was validated for parameters such as linearity, range, precision, accuracy, LOD, and LOQ.

**Result:**

The developed method adapted derivatization of gabapentin using catechol reagent measured at *λ*max 300 nm. The method used HPLC using mobile phase methanol water 50 : 50. The eluted peak of the derivatized gabapentin was separated from other used derivatization reagents. The analytical method showed to be a validated method, and all the tested validation parameters were within the accepted limits. The developed method was found to be linear (*R*^2^ = 0.9917), precise (RSD = 0.91) and accurate (% recovery = 105). Moreover, the developed method was sensitive with LOD (0.5^*∗*^10^−6^ mg/mL) and LOQ (1.5^*∗*^10^−6^ mg/mL).

**Conclusion:**

The developed method is simple and feasible with high sensitivity and selectivity. It can be applied in the analysis of gabapentin in different dosage forms and raw materials including active pharmaceutical ingredients (API). This research work can be continued in the future, and the developed method can be used for testing gabapentin in biological systems.

## 1. Introduction

Gabapentin is an antiepileptic drug with a structure analogue to *γ*-aminobutyric acid [1]. Gabapentin is approved to be used in the treatment of migraine patients as well as a prophylactic agent [1, 2]. It is also used as an anticonvulsant medication primarily used to treat partial seizures and neuropathic pain [3–5]. The recommended daily dose of gabapentin is 600-1800 mg [4]. Although gabapentin mechanism of action is not completely proven, some studies clarify its use in pain management and seizure treatment [6, 7].

Gabapentin, USP is a white to off-white crystalline powder. It is freely soluble in water, alkaline, and acidic solutions. The log of the partition coefficient (n-octanol/0.05 M phosphate buffer) at pH 7.4 is −1.25 [8, 9]. The chemical structure of gabapentin lacks chromophore, so it has a low absorption in the ultraviolet (UV) and visible range (Figure 1).

Several analytical methods were used to quantify gabapentin such as dried plasma spots [10], gas chromatography mass spectrometry (GC-MS) [11], capillary electrophoresis [12], fluorometry [13] and high-performance liquid chromatography (HPLC) [14]; US Pharmacopoeia has a monograph to analyze valproic acid using HPLC method [15].

Chemical derivitization of the analyte is widely used in recent days. The mehod is developed and used in determination of bulk or finished pharmaceutical dosage forms [16–18]. One of the derivatization analytical methods was by combining gabapentin with fluorescamine using Tecan Safire II microplate reader for recording fluorescence signal [17]. In another study, the same procedure was used, but in different pH by using borate buffer [19]. However, in a different research, gabapentin was quantified by a column that previously derivatized with 1-fluoro-2,4-dinitrobenzene as a chromatographic separation [20]. In a similar study, gabapentin was quantified with precolumn derivatization with 2,4,6-trinitrobenzenesulfonic acid by using high-performance liquid chromatography (HPLC) with UV photometric [21]. HPLC determination of gabapentin was used in different conditions by using simple automated o-phthaldialdehyde (OPA) derivatization in acidic mobile phase and fluorimetric detection [19].

A method of liquid chromatography/mass spectrometry has been developed and validated to measure gabapentin and the results were monitored for one year; a sample of protein's precipitation has been prepared with acetonitrile having internal isotopically standards with label, using reverse phase liquid chromatography ultraperformance separation with a run time of 3 minutes. Electrospray ionization in a mode of positive ion and collision-induced dissociation mass spectrometry, the analytical range was 0.1 to 100 *µ*g/mL, *R*^2^ value ranged from 0.9989 to 0.9999, the coefficient of variation and difference were less than 20% for lower limit, and as a conclusion it was a simple and cost effective method [22]. Researchers have developed and validated a sensitive gas chromatographic-mass spectrometric (GC-MS) method for gabapentin detection, Gamma-aminobutyric acid-d (2) (GABA-d(2)) was used as an internal standard during solid-phase extraction. Electrospray–ionization MS was used to check if the compound was original or not as expected 171 MW. This recommended method was used for accurate quantification of gabapentin in biological fluids for use in both pharmacokinetic and forensic studies [14].

The objective of this research is to develop a validated, simple, and feasible analytical method to quantify gabapentin in small quantities through chemical derivatization by adding a suitable conjugation to the drug chemical structure. The developed method will be validated according to the international guidelines including the international conference of harmonization and pharmacopeia [23].

## 2. Methodology

### 2.1. Reagents and Chemicals

Different reagents were used throughout the research project. All the reagents used were of analytical grade and were purchased from reliable resources, and these reagents include the following: benzoyl chloride, triethylamine, and *N, N′*-dicyclohexylcarbodiimide (DCC) were purchased form (Sigma-Aldrich, the United States. 4-Dimethylaminopyridine (DMAP) was purchased from Merck, Germany. Benzoic acid was purchased from Alfa Aesar, the United Kingdom. Dichloromethane (DCM), methanol, ammonium chloride, magnesium sulfate, and acetonitrile (ACN) were purchased from Sigma-Aldrich, Germany. Resorcinol, catechol, and hydroquinol were purchased from Sigma-Aldrich, the UK. Gabapentin was donated as a gift from Birzeit Pharmaceutical Company, Palestine.

### 2.2. Instrumentation

Different instruments were used in the project, and these instruments include magnetic stirrer-hotplate (LabTech-LMS-1003), weighing balance (Adventurer-OHAVS-AR2140), Rota evaporator (Heidolph-Rova-100), oven (UNB400–C407.0109), sonicator (MRCDC-200H), ultraviolet-visible (UV-Vis) spectrophotometer (Jenway-7315), attenuated total reflectance infrared ATR-FTIR (Thermo Fisher Nicolet IS5), shaker (Memmert, GmbH), and high-performance liquid chromatography (Waters 1525, Singapore).

### 2.3. Synthesis of Gabapentin-Dihydroxybenzene Derivatives

The conjugation was added to the gabapentin through reaction dihydroxybenzene (catechol, resorcinol, and hydroquinone). The conjugation derivatives were synthesized as shown in Figure 2:

Dihydroxybenzene (catechol/resorcinol/hydroquinone) (110.1 mg, 1 mmole) was mixed with gabapentin (171.2 mg, 1 mmole). Coupling agent EDCI 1-Ethyl-3-(3-dimethylaminopropyl) carbodiimide (191 mg, 1.23 mmoles) was then added. The reaction was evacuated from air and the reaction was allowed to run under argon gas for half an hour. 4-Dimethylaminopyridine-DMAP (122 mg, 1 mmole) was added to the mixture. The reaction was then left to stir overnight (24 h).

The reaction was monitored by TLC using mobile phase (dichloromethane 9: methanol 1). The reaction was monitored by TLC, and when it showed termination of the reaction, the reaction was quenched. The reaction mixture was rota-evaporated under reduced pressure, and the residue was purified using silica column. The mobile phase used in the purification was DCM: methanol (90 : 10). The purified compounds were used as standard later in the analytical method development.

### 2.4. Analytical Method Development

The HPLC method development was performed using coupling reaction. This particular reaction was chosen to add chromophore to the original drug (gabapentin) in order to achieve better separation and quantification. Moreover, derivatization reaction introduces chromophore to the drug acidic structure which has an extended conjugation, so it will cause a hyperchromic and bathochromic shift in the absorbance of the analyzed drug. The synthesized drug derivatives of a concentration (1 mg/mL) were scanned in the range of 200-800 nm using UV/Vis spectrophotometer. The maximum absorption was reported as *λ*max. The reaction mixture was injected in HPLC at different mobile phase compositions using mixture of solvents such as methanol, acetonitrile, and water. Other parameters like mobile and flow rates were tried at different conditions to reach the best peak shape, separation, and retention time.

### 2.5. HPLC Method Validation

The method was validated for parameters like linearity, range, accuracy, precision, LOD/LOQ, and robustness/ruggedness. Linearity and range validation parameters were performed by injecting prepared standards of different concentrations in the range of 0.5-2.5 mg/mL to the HPLC system. The area under the curve (AUC) was plotted against the concentration. The generated regression line equation along with the *R*^2^ was reported.

To evaluate the linearity and range of the method, four different test concentrations were prepared: 0.5, 1, 1.5, and 2.5 mg/1 mL. Three separate injections of each concentration were analyzed under the same conditions and the average reading was reported. The obtained peak area was plotted against the concentration; the *R*^2^ and regression line equation were recorded.

The accuracy was performed by injecting one chosen gabapentin concentration (2 mg/mL). The gabapentin was added with some widely used excipients usually used in oral dosage forms. These excipients include carboxymethyl cellulose, starch, and magnesium stearate. The percentage recovery of the test was calculated.

Instrumental precision was performed by injecting one sample (2 mg/mL) in the HPLC system five times. The RSD was then calculated for the generated AUC. Repeatability precision was established on three concentrations (0.5, 1, and 2.5 mg/mL). Three replicates of each concentration were prepared and tested; the RSD of the result was calculated.

The sensitivity of the method was established by measuring the detection limit (LOD) and the quantification limit (LOQ). One gabapentin concentration (2 mg/mL) was used to determine the limit of detection (LOD) and limit of quantification (LOQ). Serial dilutions of 10 were done to the sample, and each dilution was then injected to the HPLC system. The LOD is expressed as a concentration that gives a signal-to-noise ratio of approximately 3 : 1, while the LOQ of sample can be determined with acceptable precision and accuracy with a signal-to-noise ratio of approximately 10 : 1.

Robustness and ruggedness of the developed analytical method were performed in which the chromatographic conditions were intentionally changed slightly in order to confirm the robustness and ruggedness of the developed method. The chromatographic changes include mobile phase composition, flow rate, *λ*max, and measurement in different days. The RSD of the AUC of the generated peaks was reported.

## 3. Results and Discussion

### 3.1. Chemical Reaction

The three dihydroxybenzene molecules were reacted with the gabapentin separately under the same reaction conditions. The TLC results showed one separate spot for the derivatized gabapentin with catechol at a retention factor (Rf = 0.7), and the spot was seen on the thin layer chromatography (TLC) above the underivatized gabapentin indicating the derivatized product is more lipophilic.

The product yield of the performed reactions showed that catechol had the best yield compared to hydroquinone and resorcinol. Thus, it was decided to consider this specific reagent 1,2-dihydroxybenzene (o-dihydroxybenzene; catechol) as derivatization reagent for gabapentin in the analytical method development. The TLC result showed derivatization of gabapentin had occurred after a short time. However, full derivatization occurred only after 24 h. In order to increase the sensitivity of the method so the drug can be detected at a very low concentration, we decided to run the reaction overnight.

### 3.2. Analytical Method Development

The UV/visible scan in the range of 200-600 nm showed two *λ*max, one at 220 nm and the other was at 300 nm (Figure 3). The longer *λ*max at 300 nm was seen after adding the conjugation with an auxochrome to the original drug gabapentin which has contributed to a bathochromic and hyperchromic shift.

In the meanwhile, the underivatized gabapentin showed only one weak absorption at ***λ***max 253 nm. This result is expected as the gabapentin itself lacks the chromophore (Figure 4).

The derivatized gabapentin standard (0.2 mg/mL) along with underivatized gabapentin was run on HPLC system using the predetermined *λ*max. The generated HPLC chromatogram showed much higher absorption peak for the derivatized gabapentin than that of the underivatized one (Figure 5).

The reaction mixture was injected at different mobile phases and different HPLC conditions using different stationary phases, flow rates, and mobile phases. The best HPLC chromatographic condition used was determined when the best separation was achieved. The summarized chromatographic condition is shown in Table 1.

### 3.3. Method Validation

The developed method was validated according to the International Conference of Harmonization (ICH) and the Food and Drug Administration (FDA) [24]. Most of the validation parameters were tested and the results were within the acceptable range, which indicate the analytical method is a validated method.

Linearity and range validation parameter was done by injecting a range of standards (0.5-2.5 mg/mL) to the HPLC system. The area under the curve (AUC) was plotted against concentration. The developed method showed to be a linear relation (*R*^2^ = 0.9917); the regression line equation was found to be 3E+07x - 2E+06 (Figure 6).

The method was also evaluated for accuracy validation parameter. Gabapentin (2 mg/mL) was derivatized according the derivatization method. The AUC of generated peak was applied to the regression line equation generated from the linearity curve. The calculated concentration was found to be 2.1 mg/mL. The percentage recovery was 105%, which indicates that our developed analytical method is accurate.

Instrumental precision was done by injecting one concentration of the derivatized method (2 mg/mL) four times, and the relative standard deviation(RSD) of the area under the curve (AUC) was calculated and was found to be 0.80 which within the acceptable range. The detailed values of the individual injection are illustrated in Table 2.

Repeatability was done by preparing three concentrations of the sample (0.5, 1, and 2.5 mg/mL) which were injected in the HPLC in triplicate. The RSD was calculated for every sample concentration (0.5, 1, and 2.5 mg/mL) and was found to be 0.32, 0.91, and 0.42, respectively. The result indicates the developed method is repeatable (Table 3). Moreover, when the mean AUC of the injected concentrations was applied to the calibration curve regression line equation, the recoveries of the injected concentrations were within the acceptable range.

The method was also found to be robust under the tested variation mentioned in the methodology section; the injected concentration of gabapentin was 2 mg/mL. The result showed no variability among the generated peaks at the abovementioned condition. The RSD of the AUC was found to be 0.47 (Table 4).

The LOD and LOQ of the method are the indicators of the method sensitivity. The minimum quantity of gabapentin which the method can detect is expressed as LOD and was determined by injection diluted samples of the derivatized gabapentin. The noise-to-peak ratio (N/S) of 3 : 1 which represent the LOD was found to be 0.5^*∗*^10^−8^ mg/mL. While the noise-to-peak ratio 10 : 1 was determined as LOQ and was found to be 1.5^*∗*^10^−6^ mg/mL.

Finally, the method was found to be selective for the generated peak of the derivatized gabapentin from other reaction reagents. The peak was well separated from the other eluting peaks which have shorter retention time due to its hydrophilicity than that of the more lipophilic derivatized gabapentin. Moreover, the derivatized peak was symmetrical with an acceptable theoretical plate (Figure 7).

## 4. Conclusion

We successfully derivatized gabapentin chemically through coupling it with catechol through an ester linkage. This derivatization added conjugation to the drug. The added conjugation was utilized in analytical method development. The derivatized gabapentin is quantified at a very low concentration compared to underivatized gabapentin. The developed method was validated according to ICH and FDA guidelines. Our developed method showed high precision and accuracy and was linear. Moreover, the method showed high sensitivity and selectivity. The developed method can be applied in the analysis of drug active ingredient as a raw material and in pharmaceutical dosage form. Future work can be employed to approve the method for testing the drug in biological systems.

## Figures and Tables

**Figure 1:** Gabapentin chemical structure.

**Figure 2:** Synthetic procedure of gabapentin derivatives.

**Figure 3:** UV scan of derivatized gabapentin with catechol.

**Figure 4:** HPLC chromatogram of gabapentin.

**Figure 5:** HPLC chromatogram of chemically derivatized gabapentin.

**Figure 6:** Linearity and range.

**Figure 7:** HPLC chromatogram of chemically derivatized gabapentin in reaction mixture.

**Table 1:** Chromatographic conditions used in the HPLC system.

HPLC condition	
Λmax	300 nm
Flow rate	1 mL/minute
Mobile phase	(Methanol: Water) 50 : 50
Stationary phase	C18

**Table 2:** Instrumental precision.

Injection	AUC
1	63299501
2	64457340
3	64057764
4	64157764
5	64634758
Average	64121425.4
SD	514121.0859
RSD	0.801792977

**Table 3:** Repeatability test.

Concentration (mg/mL)	AUC
0.5	17755412
	17653532
	17749442
RSD = 0.32	

1	28957831
	28857921
	29357939
RSD = 0.91	

2.5	83217465
	83917561
	83617467
RSD = 0.42	

**Table 4:** Robustness and ruggedness test.

Condition	AUC
Analyst 1	63175584
	63571712
Analyst 2	63296473
	63342018
Flow rate 0.9 mL/min	64366812
	63366720
Flow rate 1.1 mL/min	63562420
	63456610
Mobile phase 55% water	63366810
	63499192
Mobile phase 45% water	63398281
	63942653
Wavelength 302 nm	63489294
	63933653
Wavelength 298 nm	63387594
	63476709
Average	63539533.44
SD	300227.13
RSD	0.47

## Data Availability

The data used to support the findings of this study are included within the article.

## References

[1] Goa K. L., Sorkin E. M. (1993). Gabapentin. A review of its pharmacological properties and clinical potential in epilepsy. *Drugs*.

[2] Magnus L. (1999). Nonepileptic uses of gabapentin. *Epilepsia*.

[3] Wetzel C. H., Connelly J. F. (1997). Use of gabapentin in pain management. *The Annals of Pharmacotherapy*.

[4] Goodman C. W., Brett A. S. (2019). A clinical overview of off-label use of gabapentinoid drugs. *JAMA Internal Medicine*.

[5] Attal N., Cruccu G., Baron R. (2010). EFNS guidelines on the pharmacological treatment of neuropathic pain: 2010 revision. *European Journal of Neurology*.

[6] Macdonald R. L., Kelly K. M. (1995). Antiepileptic drug mechanisms of action. *Epilepsia*.

[7] Houghton K. T., Forrest A., Awad A. (2017). Biological rationale and potential clinical use of gabapentin and pregabalin in bipolar disorder, insomnia and anxiety: protocol for a systematic review and meta-analysis. *BMJ Open*.

[8] United States Pharmacopeial C. (2011). *The United States Pharmacopeia: The National Formulary*.

[9] Chung T. C., Tai C. T., Wu H. L. (2006). Simple and sensitive liquid chromatographic method with fluorimetric detection for the analysis of gabapentin in human plasma. *Journal of Chromatography, A*.

[10] Kolocouri F., Dotsikas Y., Loukas Y. L. (2010). Dried plasma spots as an alternative sample collection technique for the quantitative LC-MS/MS determination of gabapentin. *Analytical and Bioanalytical Chemistry*.

[11] Nagaraju P., Kodali B., Datla P. V., Kovvasu S. P. (2018). LC-MS/MS quantification of tramadol and gabapentin utilizing solid phase extraction. *International journal of analytical chemistry*.

[12] Liliana Garcia L., Shihabi Z. K., Oles K. (1995). Determination of gabapentin in serum by capillary electrophoresis. *Journal of Chromatography B: Biomedical Sciences and Applications*.

[13] Zehouri J., al-Madi S., Belal F. (2001). Determination of the antiepileptics vigabatrin and gabapentin in dosage forms and biological fluids using Hantzsch reaction. *Arzneimittel-Forschung*.

[14] Lehner A. F., Stewart J., Dafalla A. (2007). Gabapentin in horses: validation of an analytical method for gabapentin quantitation. *Journal of Analytical Toxicology*.

[15] United States Pharmacopeia (2009). *Gabapentin Tablets*.

[16] Abualhasan M., Odeh N. W., Younis G. N., Zeidan O. F. (2020). Analytical method development for sodium valproate through chemical derivatization. *International journal of analytical chemistry*.

[17] Martinc B., Vovk T. (2013). A simple high-throughput method for determination of antiepileptic analogues of gamma-aminobutyric acid in pharmaceutical dosage forms using microplate fluorescence reader. *Chemical & Pharmaceutical Bulletin*.

[18] Abualhasan M. N., Watson D. G. (2019). Tagging fatty acids via choline coupling for the detection of carboxylic acid metabolites in biological samples. *Current Analytical Chemistry*.

[19] Chollet D. F., Goumaz L., Juliano C., Anderegg G. (2000). Fast isocratic high-performance liquid chromatographic assay method for the simultaneous determination of gabapentin and vigabatrin in human serum. *Journal of Chromatography B: Biomedical Sciences and Applications*.

[20] Souri E., Jalalizadeh H., Shafiee A. (2007). Optimization of an HPLC method for determination of gabapentin in dosage forms through derivatization with 1-fluoro-2, 4-dinitrobenzene. *Chemical & Pharmaceutical Bulletin*.

[21] Wad N., Kramer G. (1998). Sensitive high-performance liquid chromatographic method with fluorometric detection for the simultaneous determination of gabapentin and vigabatrin in serum and urine. *Journal of Chromatography B: Biomedical Sciences and Applications*.

[22] Palte M. J., Basu S. S., Dahlin J. L. (2018). Development and validation of an ultra-performance liquid chromatography-tandem mass spectrometry method for the concurrent measurement of gabapentin, lamotrigine, levetiracetam, monohydroxy derivative of oxcarbazepine, and zonisamide concentrations in serum in a clinical setting. *Therapeutic Drug Monitoring*.

[23] Gillings N., Todde S., Behe M. (2020). EANM guideline on the validation of analytical methods for radiopharmaceuticals. *EJNMMI radiopharmacy and chemistry*.

[24] (2022). International Conference on Harmonization. https://www.ich.org/page/quality-guidelinesInternational.

